RETRACTED

# Deleted in lymphocytic leukemia 2 induces retinoic acid receptor beta promoter methylation and mitogen activated kinase-like protein activation to enhance viability and mobility of colorectal cancer cells

**DOI:** 10.1080/21655979.2022.2076482

**Published:** 2022-05-25

**Authors:** Liang Fu, Zhitao Shi, Bingxue Chen

**Affiliations:** a Department of Anorectal Surgery, Traditional Chinese Medicine Hospital of Xinjiang Uygur Autonomous Region, Urumqi, P.R. China; b Department of General Surgery, Traditional Chinese Medicine Hospital of Xinjiang Uygur Autonomous Region, Urumqi. P.R. China; c Department of General Surgery, Changzhou No. 2 Peoples’ Hospital, Changzhou, P.R. China

**Keywords:** LncRNA DLEU2, DNA methylation, RARB, MAPK, colorectal cancer

## Abstract

Abnormal expression of long non-coding RNAs (lncRNAs) is frequently linked to the pathogenesis of colorectal cancer (CRC). This work explored the function of lncRNA deleted in lymphocytic leukemia 2 (DLEU2) in CRC and the epigenetic mechanism. Candidate oncogenes in CRC were predicted using a GSE146587 dataset. DLEU2 was highly expressed in CRC according to the bioinformatic analysis and its high expression was detected in CRC cells compared to the normal colon epithelial cells (FHC). Downregulation of DLEU2 in CRC SW480 and HT29 cells suppressed viability, migration, invasiveness, and resistance to apoptosis of cells. The mRNA microarray analysis was performed to explore the key molecules mediated by DLEU2. Retinoic acid receptor beta (RARB) expression was elevated in cells after DLEU2 downregulation. The promoter methylation of RARB was enhanced in CRC cells compared to normal FHC cells. DLEU2 induced promoter methylation of RARB to downregulate its expression. Further silencing of RARB restored proliferation and invasiveness of cells blocked by sh-DLEU2. Upregulation of DLEU2 activated the mitogen activated kinase-like protein (MAPK) signaling pathway to trigger CRC progression. In conclusion, this study demonstrates that DLEU2 enhances viability and mobility of CRC cells by inducing RARB promoter methylation and activating the MAPK signaling pathway.

## Highlights

- DLEU2 expression is increased in CRC.
- Silencing of DLEU2 suppresses proliferation and invasiveness of CRC cells.
- RARB expression is increased in CRC cells after DLEU2 silencing.
- DLEU2 recruits DNMT1 to induce RARB DNA methylation.
- DLEU2 reduces RARB expression to inactivate the MAPK signaling pathway.

## Introduction

Colorectal cancer (CRC) represents the third most prevailing cancer and the fourth leading cause of cancer-related death [1]. Aging, genetic, and environmental factors are major risk factors implicated in the development of CRC [2], other factors including alcohol and tobacco consumption and bad dietary habits may also play a role [3,4]. Thanks to effective screening measures, prompt interventions, and improved treatment strategies, mortality from CRC has declined by approximately 35% from 1990 to 2007 and about 50% from the peak [5]. However, there were about 1.8 million new CRC cases in 2018 and 881,000 people died from this malignancy [6,7]. In addition, the decline in overall mortality might have masked the mortality rate for young adult patients since the death rate has increased from 3.9 per 100,000 in 2004 to 4.3 per 100,000 in 2014 among young populations [2]. Therefore, management of CRC remains a considerable challenge for the health-care administrations and the whole society.

RETRACTED

Epigenetics is a study of inherited changes in gene expression of phenotype that do not involve DNA sequence alterations [8]. The major epigenetic mechanisms include histone modifications and DNA methylation, and the epigenetic regulations by non-coding RNAs (ncRNAs) play a critical role in cell growth, differentiation, and cancer [8]. Long ncRNAs (lncRNAs), defined as ncRNA molecules over 200 nucleotides long, have been emergingly concerned because their aberrant expression is frequently correlated with the development of human cancers [9]. For instance, LINC00857 and LINC00997 have recently been demonstrated to promote the carcinogenesis of CRC by interacting with other RNA molecules [10,11]. Advanced bioinformatics systems and tools have offered great convenience and opportunity for the screening of crucial molecular factors linked to the progression of CRC [12]. We identified lncRNA deleted in lymphocytic leukemia 2 (DLEU2) as an aberrantly expressed gene in CRC by bioinformatics analysis. DLEU2 has been associated with the proliferation and invasiveness of CRC cells [13], yet the possible molecules involved remain largely unknown. Intriguingly, certain lncRNAs may serve as manipulators for DNA methylation by regulating specific DNA methyltransferases (DNMTs) or Ten-eleven translocation family of enzymes [14,15]. DNA methylation refers to the selective methylation of cytosine within a cytosine-phosphate-guanine (CpG) dinucleotide, thus forming 5-methylcytosine [16,17]. In general, methylation of CpG Islands can stably silence gene expression by recruiting suppressive methyl-binding proteins and blocking transcription factor binding [18]. Importantly, our microarray analysis suggested that retinoic acid receptor beta (RARB) gene was inversely associated with DLEU2 expression in CRC cells. Hypermethylation and the downregulation of RARB has been found in high-grade cancers and linked to tumor progression [19,20].

RETRACTED

Taken together, we hypothesized that DLEU2 possibly regulates promoter DNA methylation of RARB to induce gene silencing and trigger the development of CRC. The regulation of DLEU2 on RARB was analyzed by detecting expression. The involvement of specific DNMTs in the regulation of DNA methylation was analyzed by immunoprecipitation assays. The functions of DLEU2 and RARB in the proliferation, migration, and invasiveness of the CRC cells were analyzed by gain- and loss-of-function assays. We also identified correlation of RARB with the mitogen activated kinase-like protein (MAPK) signaling pathway in CRC progression.

## Material and methods

### Cells

CRC cell lines SW620 (CCL-227), SW480 (CCL-228), HT29 (HTB-38), LOVO (CCL-229), and HCT116 (CCL-247), and a normal colon epithelial cell line FHC (CRL-1831) were procured from American Type Culture Collection (Manassas, VA, USA). FHC cells were cultured in minimum essential medium, and the CRC cells were cultured in Roswell Park Memorial Institute-1640. All media were procured from Thermo Fisher Scientific Inc. (Waltham, MA, USA) and added with 10% fetal bovine serum (FBS) and 1% penicillin/streptomycin. The culture condition was maintained at 37°C with 5% CO_2._

### Cell transfection and treatment

Short hairpin (sh) RNA of DLEU2 (5ʹ-GAAGAAATGCCAACTGCTTGA-3ʹ), sh-RARB (5ʹ-ACACTTGTCACCGAGATAAGAACTGTGTTATTAATAAAGTC-3ʹ), sh-negative control (NC), and the pcDNA 3.1 plasmid overexpressing DLEU2 were synthesized and provided by Vectorbuilder Co., Ltd. (Guangdong, China). The shRNAs or pcDNAs were transfected into cells following the instructions of Lipofectamine 2000 (Thermo Fisher Scientific). After 48 h, the stably transfected cells were screened by puromycin (2 μg/mL) for subsequent use. Thereafter, morphologic changes of cells were observed and captured under an optical microscope (Nikon Corporation, Tokyo, Japan). The dimethyl sulfoxide (DMSO) and 5-aZa-CDR (CAS No. 2353–33-5), a DNA methylation inhibitor, were procured from Sigma-Aldrich (Merck KGaA, Darmstadt, Germany). Cells were treated with 5 μM 5-aZa-CDR dissolved in DMSO for 24 h to suppress DNA methylation [21]. Moreover, cells were treated with 1 μM Dehydrocorydaline (HY-N0674, MedChemExpress [MCE], Monmouth Junction, NJ, USA), p38-specific agonist, for 24 h to activate the p38/MAPK signaling pathway [22]. Cells treated with equal volume of DMSO were set to controls.

### Reverse transcription quantitative polymerase chain reaction (RT-qPCR)

RNA was extracted from cells and tissues using the TRIzol reagent (Thermo Fisher Scientific) and examined by a spectrophotometer. Thereafter, the RNA was reverse-transcribed to cDNA using a cDNA synthesis kit (Takara Holdings Inc., Kyoto, Japan). The PCR system was configured and amplified using the SYBR RT-qPCR kit (Thermo Fisher Scientific). The primers are listed in Table 1. Glyceraldehyde-3-phosphate dehydrogenase (GAPDH) served as the internal loading for the measurement of DLEU2 and RARB mRNA. Gene expression values were evaluated by the 2^−ΔΔCt^ method [23].

RETRACTED

**Table 1.** Primer sequences for RT-qPCR

Primers	Sequence (5’-3’)
DLEU2	F: TGAAGATGTCTTTTGAAAGGTGTAC
	R: ACTTTTTCCATGAGGAGGTACAGT
RARB	F: GGTTTCACTGGCTTGACCATCG
	R: CCGTCTGAGAAAGTCATGGTGTC
GAPDH	F: GTCTCCTCTGACTTCAACAGCG
	R: ACCACCCTGTTGCTGTAGCCAA
U6	F: CTCGCTTCGGCAGCACAT
	R: TTTGCGTGTCATCCTTGCG
18S	F: ACCCGTTGAACCCCATTCGTGA
	R: GCCTCACTAAACCATCCAATCGG

Note: RT-qPCR, reverse transcription quantitative polymerase chain reaction; DLEU2, deleted in lymphocytic leukemia 2; RARB, retinoic acid receptor beta; GAPDH, glyceraldehyde-3-phosphate dehydrogenase.

### Immunoblot analysis

Cells were lysed in radio-immunoprecipitation assay lysis buffer on ice to extract total protein. The protein concentration was evaluated using the enhanced bicinchoninic acid kit (Beyotime Biotechnology Co. Ltd., Shanghai, China). An equal amount of protein was run on 10% sodium dodecyl sulfate-polyacrylamide gel electrophoresis and transferred on polyvinylidene fluoride membranes. The membranes were soaked in nonfat milk for 2 h to block the nonspecific binding sites and then reacted with the primary antibodies at 4°C overnight, and then with horseradish peroxidase (HRP)-conjugated secondary antibody (1:2,000, ab205718, Abcam Inc., Cambridge, MA, USA) at 25°C for 1 h. The blot bands were developed using the enhanced chemiluminescence kit (Thermo Fisher Scientific). Relative protein expression was evaluated using the Image J software. The primary antibodies were anti-RARB (1:1,000, GTX66626, GeneTex, CA, USA), anti-pRaf (Ser299) (1:1,000, #4431S, Cell Signaling Technology (CST), Beverly, MA, USA), anti-Raf (1:1,000, #4432S, CST), anti-p-p38 (1:2,000, GTX133460, GeneTex), anti-p38 (1:1,000, GTX110720, CST), anti-p-ERK1/2 (1:1,000, ab201015, Abcam), anti-ERK1/2 (1:10,000, ab184699, Abcam), and anti-GAPDH (1:10,000, ab181603, Abcam) [24].

### Cell counting kit-8 (CCK-8) method

Stably transfected SW480 and HT29 cells were digested in 0.02% ethylene diamine tetraacetic acid-0.25% trypsin to prepare cell suspension. Cells were seeded in 96-well plates at 3,000 cells per well and cultured at 37°C with 5% CO_2_. At the 0, 24, 48, and 72 h, respectively, 10 μL CCK-8 reagent (MCE) was added to each well. After another 2 h of culture, the optical density at 450 nm of each well was read to evaluate viability of cells [25].

RETRACTED

### Transwell assay

The 24-well Transwell chambers (8 μm in diameter, Corning, NY, USA) were used to examine the migration and invasiveness of the SW480 and HT29 cells. For invasiveness detection, stably transfected SW480 or HT29 cells (1 × 10^5^) were dispersed in 200 μL serum-free medium and loaded into the apical chambers precoated with Matrigel. The basolateral chambers were filled with 600 μL 10% FBS-supplemented medium. Migration ability of cells was examined likewise except for the Matrigel precoating on the apical chambers. After 48 h, the invasive or migratory cells were fixed in 4% paraformaldehyde (PFA) and stained with 0.5% crystal violet for 20 min. The numbers of invasive or migratory cells were calculated under the light microscope [26].

### Flow cytometry

Apoptosis of cells was determined following the protocol of an Annexin V-fluorescein isothiocyanate detection kit (Thermo Fisher Scientific). In short, after digestion, the cells were incubated with fluorescein isothiocyanate and propidium iodide avoiding light exposure at 23°C for 15 min. The cell apoptosis was then examined utilizing a flow cytometer (BD Biosciences, Franklin Lakes, NJ, USA) and the apoptosis rate was analyzed by the Flow Jo software [27].

### Subcellular localization of DLEU2

Subcellular localization of DLEU2 in SW480 and HT29 cells was first determined using a fluorescence in situ hybridization (FISH) assay. Well growing cells (5 × 10^5^/mL) were fixed in 4% PFA for 30 min. The cells were washed and incubated with protease K, dehydrated in an increasing series of alcohol, and hybridized with fluorescence-labeled DLEU2 probe. The nuclei were stained by 4’, 6-diamidino-2-phenylindole (Life Technologies, CA, USA). The fluorescence was observed under the microscope [28]. In addition, the nuclear- and cytoplasmic-RNA was separated according to the instruction manual of a PARIS^TM^ kit (Thermo Fisher Scientific). Expression of the nuclear- and cytoplasmic-RNA was then examined using RT-qPCR to examine the distribution of DLEU2 in cells [29].

### Microarray analysis

Microarray analysis was performed utilizing the Agilent Array platform (Agilent Technologies, Santa Clara, CA, USA). Samples were prepared and microarray was hybridized following the manufacturer’s instruction manual. Total RNA from HT29 cells with DLEU2 knockdown was extracted using the TRIzol again. The mRNA from total RNA was isolated using a GenElute™ Direct mRNA preparation kit (DMN70, Sigma-Aldrich). The mRNA was purified and hybridized with the microarray chips. After that, the microarray chips were scanned using the GenePix 4000B scanner (Axon Instruments, Foster City, CA, USA). The microarray chip images were analyzed using the Agilent Feature Extraction software (Agilent Technologies). The data were processed and analyzed using the GeneSpring GX v12.0 software (Agilent Technologies) [30].

RETRACTED

### Quantitative methylation specific PCR (qMSP)

A Genomic DNA Kit (TianGen Biotech Co., Ltd., Beijing, China) was used to obtain human genomic DNA from cells, which was subjected to bisulfite modification using a DNA methylation kit (Zymo Research, Orange, CA, USA). The PCR product was examined by qPCR. The MSP primers of the CpG Island of RARB promoter were designed via MethPrimer (http://www.urogene.org/cgi-bin/methprimer/methprimer.cgi) [31]. The primer sequences are shown in Table 2.

**Table 2.** Primer sequences for qMSP

CpG sites	Primers	Sequences	
Set1	methylated-specific primer	Left	GTGTTTAACGTGAGTTAGGAGTAGC
		Right	AACCAAAAAAACAAACAACGAA
	unmethylated-specific primer	Left	TGGTGTTTAATGTGAGTTAGGAGTAGT
		Right	AAACAACCAAAAAAACAAACAACA
Set2	methylated-specific primer	Left	GTGTTTAACGTGAGTTAGGAGTAGC
		Right	AACCAAAAAAACAAACAACGAA
	unmethylated-specific primer	Left	TGGTGTTTAATGTGAGTTAGGAGTAGT
		Right	ACAACCAAAAAAACAAACAACAAA
Set3	methylated-specific primer	Left	GTGTTTAACGTGAGTTAGGAGTAGC
		Right	AACCAAAAAAACAAACAACGAA
	unmethylated-specific primer	Left	TGGTGTTTAATGTGAGTTAGGAGTAGT
		Right	AACAACCAAAAAAACAAACAACAA
Set4	methylated-specific primer	Left	GTGTTTAACGTGAGTTAGGAGTAGC
		Right	CAACCAAAAAAACAAACAACGA
	unmethylated-specific primer	Left	TGGTGTTTAATGTGAGTTAGGAGTAGT
		Right	ACAACCAAAAAAACAAACAACAAA
Set5	methylated-specific primer	Left	GTGTTTAACGTGAGTTAGGAGTAGC
		Right	CAACCAAAAAAACAAACAACGA
	unmethylated-specific primer	Left	TGGTGTTTAATGTGAGTTAGGAGTAGT
		Right	AAACAACCAAAAAAACAAACAACA

Note: QMSP, quantitative methylation specific polymerase chain reaction; CpG, cytosine-phosphate-guanine.

### RNA immunoprecipitation (RIP) assay

Binding relationship between DLEU2 and DNMT1 was examined using the Imprint® RIP kit (RIP-12RXN, Sigma-Aldrich). In short, the SW480 and HT29 cells were digested and resuspended, and incubated in formaldehyde at ~23°C for 10 min for RNA-protein crosslinking, which was terminated by glycine. The cells were lysed thereafter and centrifuged at 4,500 *g* to collect the supernatant, to which the magnetic beads-conjugated with anti-DNMT1 (1:100, ab92314, Abcam) were added for overnight incubation at 4°C. After that, the beads were washed with IP lysis buffer and incubated with RIP buffer at 65°C for 1 h for de-crosslinking. The DLEU2 expression in the extracted was examined by RT-qPCR as mentioned above [32].

### Chromatin immunoprecipitation (ChIP)-qPCR

A Pierce™ magnetic ChIP kit (26,157, Thermo Fisher Scientific) was used to analyze the binding between DNMT1 and RARB promoter. In short, the CRC cells were seeded in six-well plates and treated with 1% formaldehyde for 30 min for DNA-protein cross-linking. After termination by formaldehyde, the cells were washed and ultrasonicated, and then centrifuged at 4°C at 4,500 *g* for 5 min to collect the supernatant, to which the magnetic beads-conjugated with anti-DNMT1 (1:100, ab92314, Abcam) were added for overnight incubation at 4°C. The beads were washed and centrifuged at 2,000 g for 1 min. The precipitated complexes were washed and treated with 5 M NaCl at 65°C for 5 h for de-crosslinking. The RARB DNA fragments were analyzed by qPCR analysis.

RETRACTED

### Statistical analysis

SPSS 22.0 (IBM Corp. Armonk, NY, USA) was used for data analysis. Measurement data from at least three repetitions were expressed as the mean ± standard deviation. Differences were analyzed by the one- or two-way analysis of variance (ANOVA) followed by Tukey’s multiple comparisons. Statistically significant difference was set at *p* < 0.05.

## Results

### Starting paragraph

Our preliminary bioinformatics analyses predicted DLEU2 as an aberrantly expressed lncRNA in CRC, and RARB was analyzed as a candidate downstream target mediated by DLEU2. As lncRNAs have been reported with the capacity of manipulating DNA methylation, which is usually correlated with gene suppression, we hypothesized that DLEU2 might recruit specific DNMTs to induce DNA methylation and transcriptional suppression of RARB. We analyzed the interactions between DLEU2, DNMT1, and RARB via immunoprecipitation assays and analyzed the roles of DLEU2 and RARB in the proliferation, migration, and invasiveness of two CRC cells SW480 and HT29 by gain- and loss-of-function assays. The involvement of MAPK signaling in the DLEU2/RARB cascade-mediated CRC progression was examined by rescue experiments using a p38-specific agonist Dehydrocorydaline in cells.

### DLEU2 expression is elevated in CRC

To explore the potential genes involved in the carcinogenesis of CRC, we analyzed three CRC-related gene expression datasets GSE146587, GSE156720, and GSE184093 from Gene Expression Omnibus (GEO, https://www.ncbi.nlm.nih.gov/gds/?) to obtain genes with aberrant expression in CRC. The volcano plots are presented in Figure 1a. We obtained four lncRNAs including colorectal neoplasia differentially expressed (CRNDE), LINC00460, Pvt1 oncogene (PVT1), and DLEU2 (Figure 1b) that were commonly dysregulated in the three datasets. Among the four candidate genes, the role of DLEU2 in CRC and the molecules are relatively less studied. We therefore chose DLEU2 as the subject of this work. Data in the Gene Expression Profiling Interactive Analysis (GEPIA) system (http://gepia.cancer-pku.cn/detail.php) suggested that DLEU2 was expressed at high levels in a multitude of cancers (Figure 1c). This is also true for patients with CRC compared to healthy individuals (Figure 1d). Thereafter, we examined the DLEU2 expression in the CRC cells. Importantly, DLEU2 was expressed at high levels in all CRC cell lines (SW620, SW480, HT29, LOVO, and HCT116) versus the normal FHC cells (Figure 1e) (SW620 vs. FHC: *p* = 0.0041; SW480 vs. FHC: *p* < 0.0001; HT29 vs. FHC: *p* < 0.0001; LOVO vs. FHC: *p* = 0.0251; HCT116 vs. FHC: *p* = 0.0003). The HT29 and SW480 cells showing relatively high DLEU2 levels were selected for subsequent experiments.

RETRACTED

**Figure 1.** DLEU2 expression is increased in CRC. (a) volcano plots for differentially expressed genes between CRC and normal colorectal tissues screened using three GEO datasets GSE146587, GSE156720, and GSE184093; (b) common lncRNAs with differential expression in three datasets compared by a Venn diagram; (c) expression of DLEU2 in multiple cancer types in GEPIA (see full text of the cancer types in Supplementary Table 1); (d) DLEU2 expression in patients with CRC (COAD, colon adenocarcinoma) and healthy individuals in GEPIA; (e) DLEU2 expression in CRC cell lines (SW620, SW480, HT29, LOVO and HCT116) and in normal FHC cells determined by RT-qPCR (one-way ANOVA) (SW620 vs. FHC: *p* = 0.0041; SW480 vs. FHC: *p* < 0.0001; HT29 vs. FHC: *p* < 0.0001; LOVO vs. FHC: *p* = 0.0251; HCT116 vs. FHC: *p* = 0.0003). Repetition = 3.

### Silencing of DLEU2 suppresses proliferation and invasiveness of CRC cells

ShRNA silencing of DLEU2 was introduced in SW480 and HT29 cells (Figure 2a) (SW480: *p* = 0.0001; HT29: *p* = 0.0004). It was found that the shape of CRC cells was changed from normal to round after stable transfection of sh-DLEU2 (Figure 2b). Thereafter, the activity of cells was examined. The CCK-8 method showed that the viability of cells was significantly decreased after DLEU2 knockdown (Figure 2c) (SW480: 0 h, *p* = 0.9996; 24 h, *p* = 0.2507; 48 h, *p* = 0.0012; 72 h, *p* < 0.0001; HT29: 0 h, *p* = 0.9963; 24 h, *p* = 0.2023; 48 h, *p* = 0.0006; 72 h, *p* < 0.0001). Transwell assays showed that the counts of cells migrated to (Figure 2d) (SW480: *p* < 0.0001; HT29: *p* < 0.0001) or invaded (Figure 2e) (SW480: *p* = 0.0001; HT29: *p* = 0.0003) the lower membranes were reduced after DLEU2 silencing. Moreover, the apoptosis of SW480 and HT29 cells was increased by sh-DLEU2 (figure 2f) (SW480: *p* < 0.0001; HT29: *p* < 0.0001). These results demonstrate that silencing of DLEU2 suppresses proliferation and invasiveness of CRC cells.

RETRACTED

**Figure 2.** DLEU2 silencing suppresses proliferation and invasiveness of CRC cells. (a) DLEU2 expression in SW480 and HT29 cells after sh-DLEU2 transfection determined by RT-qPCR (two-way ANOVA) (SW480: *p* = 0.0001; HT29: *p* = 0.0003); (b) morphologic changes in SW480 and HT29 cells after sh-DLEU2 transfection; (c) viability of SW480 and HT29 cells determined by the CCK-8 method (two-way ANOVA) (SW480: 0 h, *p* = 0.9996; 24 h, *p* = 0.2507; 48 h, *p* = 0.0012; 72 h, *p* < 0.0001; HT29: 0 h, *p* = 0.9963; 24 h, *p* = 0.2023; 48 h, *p* = 0.0006; 72 h, *p* < 0.0001); (d-e), migration (d) and invasiveness (e) of SW480 and HT29 cells analyzed by Transwell assays (two-way ANOVA) (D: migration: SW480: *p* < 0.0001; HT29: *p* < 0.0001; E: invasiveness: SW480: *p* = 0.0001; HT29: *p* = 0.0003); (f) apoptosis of SW480 and HT29 cells detected by flow cytometry (two-way ANOVA) (SW480: *p* < 0.0001; HT29: *p* < 0.0001). Repetition = 3.

### RARB expression is elevated in CRC cells after DLEU2 silencing

To explore the downstream molecules, we first explored the sub-cellular distribution of DLEU2. The nuclear-cytoplasmic RNA separation and FISH assays suggested that DLEU2 was mainly distributed in nucleus in SW480 and HT29 cells (Figure 3a-b). Next, the mRNA microarray analysis suggested that the RARB mRNA was significantly upregulated in HT29 cells transfected with sh-DLEU2 (Figure 3c). According to the data in the Cancer Genome Atlas (TCGA), RARB showed a universal poor expression in multiple cancers (Figure 3d). Data in GEPIA also showed that RARB was poorly expressed in patients with CRC compared to the healthy populations (Figure 3e). Thereafter, the RT-qPCR and immunoblot assays indicated that the mRNA (figure 3f) and protein (Figure 3g) levels of RARB in SW480 and HT29 cells were significantly elevated upon DLEU2 silencing (G: SW480: *p* < 0.0001; HT29: *p* < 0.0001; H, SW480: *p* < 0.0001; HT29: *p* = 0.0001).

**Figure 3.** RARB expression is elevated in CRC cells after DLEU2 silencing. (a-b), sub-cellular localization of DLEU2 in SW480 and HT29 cells examined by nuclear- and cytoplasmic-RNA separation (a) and FISH (b) assays; (c), differentially expressed mRNAs between HT29 cells transfected with sh-DLEU2 or sh-NC examined by microarray analysis; (d), RARB expression in cancers in TCGA; (e) RARB expression in patients with CRC (COAD) and healthy populations in GEPIA database; (f-g) mRNA (f) (SW480: *p* < 0.0001; HT29: *p* < 0.0001) and protein (g) (SW480: *p* < 0.0001; HT29: *p* = 0.0001) levels of RARB in DLEU2-silencing SW480 and HT29 cells examined by RT-qPCR and immunoblot analysis (two-way ANOVA). Repetition = 3.

RETRACTED

### High cin RARB promoter in CRC cells

Hypermethylation-induced inactivation of tumor-suppressing cells is a frequent event involved in tumorigenesis. To evaluate if there is a methylation modification in the promoter of RARB that leads to RARB downregulation, we first obtained the CpG Island sequence at the RARB promoter (Figure 4a). The accuracy of the CpG Island sequences was confirmed by MethPrimer, and five sequences (Set1, Set2, Set3, Set4, and Set5) were obtained (Figure 4b). Next, we examined the DNA methylation level in RARB promoter in SW480, HT29, and FHC cells. Compared to that in FHC cells, the methylation level at the Set2 sites in RARB promoter was significantly elevated in SW480 and HT29 cells, whereas the methylation level at other sites showed no significant changes (Figure 4c) (Set1: SW480 vs. FHC: *p* = 0.7177; HT29 vs. FHC: *p* = 0.8936; Set2: SW480 vs. FHC: *p* = 0.0004; HT29 vs. FHC: *p* = 0.0002; Set3: SW480 vs. FHC: *p* = 0.9702; HT29 vs. FHC: *p* = 0.9213; Set4: SW480 vs. FHC: *p* = 0.9865, HT29 vs. FHC: *p* = 0.9648; Set5: SW480 vs. FHC: *p* = 0.9702, HT29 vs. FHC: *p* = 0.9966). Subsequently, the RIP assay found that the DLEU2 could bind to DNMT1 (Figure 4d) (SW480: *p* < 0.0001; HT29: *p* < 0.0001). Moreover, the ChIP assay revealed that a large number of RARB promoter fragments were enriched by anti-DNMT1 (Figure 4e) (SW480: *p* < 0.0001; HT29: *p* < 0.0001). These results reveal that DLEU2 recruit DNMT1 to the promoter of RARB to induce its DNA methylation. The CRC cells were treated with 5-aZa-CDR, after which the methylation level in the RARB promoter was significantly reduced (figure 4f) (SW480: *p* < 0.0001; HT29: *p* < 0.0001). In this setting, the mRNA and protein levels of RARB were significantly elevated (Figure 4g-h) (G: SW480: *p* < 0.0001; HT29: *p* < 0.0001; H: SW480: *p* < 0.0001; HT29: *p* = 0.0001). Collectively, these results suggest that DNA hypermethylation in the RARB promoter is a major cause for its poor expression in CRC cells.

**Figure 4.** High DNA methylation level is identified in RARB promoter in CRC cells. (a) information of the CpG Island sequence at the RARB promoter obtained from NCBI; (b) validation of the CpG Island sequence; (c) DNA methylation level at different CpG Island sites in the RARB promoter in SW480, HT29 and FHC cells examined by qMSP (one-way ANOVA, compared to FHC cells) (Set1: SW480 vs. FHC: *p* = 0.7177; HT29 vs. FHC: *p* = 0.8936; Set2: SW480 vs. FHC: *p* = 0.0004; HT29 vs. FHC: *p* = 0.0002; Set3: SW480 vs. FHC: *p* = 0.9702; HT29 vs. FHC: *p* = 0.9213; Set4: SW480 vs. FHC: *p* = 0.9865, HT29 vs. FHC: *p* = 0.9648; Set5: SW480 vs. FHC: *p* = 0.9702, HT29 vs. FHC: *p* = 0.9966); (d) binding between DNMT1 and DLEU2 examined by RIP assay (two-way ANOVA) (SW480: *p* < 0.0001; HT29: *p* < 0.0001); (e) binding relationship between DNMT1 and RARB promoter examined by ChIP-qPCR assay (two-way ANOVA) (SW480: *p* < 0.0001; HT29: *p* < 0.0001); (f) DNA methylation level of RARB in SW480 and HT29 cells after 5-aZa-CDR treatment examined by qMSP (two-way ANOVA) (SW480: *p* < 0.0001; HT29: *p* < 0.0001); (g-h). mRNA (g) (SW480: *p* < 0.0001; HT29: *p* < 0.0001) and protein (h) (SW480: *p* < 0.0001; HT29: *p* = 0.0001) levels of SW480 and HT29 cells after 5-aZa-CDR treatment examined by RT-qPCR and immunoblot analysis (two-way ANOVA). Data were collected from three independent experiments. Repetition = 3. *p < 0.05; **p < 0.01.

RETRACTED

### DLEU2 activates the MAPK signaling pathway by enhancing RARB promoter methylation

We next explored the downstream molecules mediated by RARB. The downstream genes of RARB were analyzed by a Kyoto Encyclopedia of Genes and Genomes (KEGG) analysis and those genes showed an over 0.5 correlation coefficient with RARB were visualized using a bubble chart. The bubble chart included top 12 correlated signaling pathways, and the RARB targets were largely enriched in the MAPK signaling (Figure 5a-b). Later, oe-DLEU2 and sh-DLEU2 were administrated in SW480 and HT29 cells. It was observed that oe-DLEU2 elevated DLEU2 whereas reduced RARB mRNA expression. By contrast, sh-DLEU2 led to decreased DLUE2 expression whereas elevated RARB expression (Figure 5c) (DLEU2: SW480: oe-DLEU2 vs. NC: *p* < 0.0001; sh-DLEU2 vs. NC: *p* = 0.0025; HT29: oe-DLEU2 vs. NC: *p* < 0.0001; sh-DLEU2 vs. NC. *p* = 0.0087; RARB: SW480: oe-DLEU2 vs. NC: *p* = 0.0024, sh-DLEU2 vs. NC: *p* < 0.0001; HT29: oe-DLEU2 vs. NC: *p* = 0.001, sh-DLEU2 vs. NC: *p* < 0.0001). It was indicated that DLEU2 overexpression increased DNA methylation in the RARB promoter, but downregulation of DLEU2 led to inverse trends (Figure 5d) (SW480: oe-DLEU2 vs. NC: *p* < 0.0001, sh-DLEU2 vs. NC *p* = 0.0013; HT29: oe-DLEU2 vs. NC *p* < 0.0001, sh-DLEU2 vs. NC: *p* = 0.0033). After that, we determined the activity of the MAPK pathway in cells. It was found that overexpression of DLEU2 increased phosphorylation of the Raf, p38, and ERK, but the phosphorylation extent of the Raf, p38, and ERK was reduced by sh-DLEU2 (Figure 5e) (see *p* values in Table 3). However, the total protein levels of Raf, p38, and ERK were not affected upon DLEU2 alterations.

**Figure 5.** DLEU2 activates the MAPK-signaling pathway via enhancing RARB promoter methylation. (a-b) target genes of RARB showing an over 0.5 correlation coefficient with RARB and the KEGG pathway analysis based on these genes; (c) RARB expression in cells after oe-DLEU2 or sh-DLEU2 transfections detected by RT-qPCR (two-way ANOVA) (DLEU2: SW480: oe-DLEU2 vs. NC: *p* < 0.0001; sh-DLEU2 vs. NC: *p* = 0.0025; HT29: oe-DLEU2 vs. NC: *p* < 0.0001; sh-DLEU2 vs. NC. *p* = 0.0087; RARB: SW480: oe-DLEU2 vs. NC: *p* = 0.0024, sh-DLEU2 vs. NC: *p* < 0.0001; HT29: oe-DLEU2 vs. NC: *p* = 0.001, sh-DLEU2 vs. NC: *p* < 0.0001); (d) methylation level in the RARB promoter examined by qMSP (two-way ANOVA) (SW480: oe-DLEU2 vs. NC: *p* < 0.0001, sh-DLEU2 vs. NC *p* = 0.0013; HT29: oe-DLEU2 vs. NC *p* < 0.0001, sh-DLEU2 vs. NC: *p* = 0.0033); (e) phosphorylation and protein levels of Raf, p38, and ERK in CRC cells determined by immunoblot analysis (two-way ANOVA) (see *p* values in Table 3). Repetition = 3.

RETRACTED

**Table 3.** *P* values of the phosphorylation extent of the Raf, p38, and ERK between the oe-DLEU2 and NC groups in SW480 and HT29 cells

Cell lines	Protein	Data comparisons	*P* values
SW480	p-Raf	oe-DLEU2 vs. NC	*p* = 0.0008
		sh-DLEU2 vs. NC	*p* = 0.0278
	Raf	oe-DLEU2 vs. NC	*p* = 0.9725
		sh-DLEU2 vs. NC	*p* = 0.9368
	p-p38	oe-DLEU2 vs. NC	*p* = 0.005
		sh-DLEU2 vs. NC	*p* = 0.016
	p38	oe-DLEU2 vs. NC	*p* = 0.8948
		sh-DLEU2 vs. NC	*p* = 0.8527
	p-ERK	oe-DLEU2 vs. NC	*p* = 0.0027
		sh-DLEU2 vs. NC	*p* = 0.0032
	ERK	oe-DLEU2 vs. NC	*p* = 0.9725
		sh-DLEU2 vs. NC	*p* = 0.9725
HT29	p-Raf	oe-DLEU2 vs. NC	*p* = 0.0044
		sh-DLEU2 vs. NC	*p* = 0.0136
	Raf	oe-DLEU2 vs. NC	*p* = 0.9752
		sh-DLEU2 vs. NC	*p* = 0.7988
	p-p38	oe-DLEU2 vs. NC	*p* = 0.023
		sh-DLEU2 vs. NC	*p* = 0.0078
	p38	oe-DLEU2 vs. NC	*p* = 0.9046
		sh-DLEU2 vs. NC	*p* > 0.9999
	p-ERK	oe-DLEU2 vs. NC	*p* = 0.0078
		sh-DLEU2 vs. NC	*p* = 0.023
	ERK	oe-DLEU2 vs. NC	*p* = 0.7988
		sh-DLEU2 vs. NC	*p* = 0.9046

### Silencing of RARB blocks the inhibiting role of sh-DLEU2 in CRC cells

To validate if RARB is a downstream functional target of DLEU2, sh-RARB or sh-NC was additionally transfected into SW480 and HT29 cells after sh-DLEU2 transfection, and the successful knockdown was detected by RT-qPCR (Figure 6a) (DLEU2: SW480: sh-DLEU2 + sh-NC vs. sh-DLEU2 + sh-RARB: *p* = 0.9657; HT29: sh-DLEU2 + sh-NC vs. sh-DLEU2 + sh-RARB: *p* = 0.8714; RARB: SW480: sh-DLEU2 + sh-NC vs. sh-DLEU2 + sh-RARB: *p* = 0.0006; HT29: sh-DLEU2 + sh-NC vs. sh-DLEU2 + sh-RARB: *p* = 0.0001). It was found that the viability of CRC cells, which was initially suppressed by sh-DLEU2, was restored after further RARB silencing (Figure 6b) (SW480: 0 h: *p* = 0.9931; 24 h: *p* = 0.4837; 48 h: *p* = 0.0069; 72 h: *p* = 0.0001; HT29: 0 h: *p* = 0.9947; 24 h: *p* = 0.2835; 48 h *p* = 0.0013; 72 h: *p* < 0.0001). In addition, the migration and invasiveness of cells within 48 h were increased after RARB silencing (Figure 6c-d) (C: SW480: sh-DLEU2 + sh-NC vs. sh-DLEU2 + sh-RARB: *p* = 0.0005; HT29: sh-DLEU2 + sh-NC vs. sh-DLEU2 + sh-RARB *p* = 0.0002; D: SW480: sh-DLEU2 + sh-NC vs. sh-DLEU2 + sh-RARB: *p* = 0.001; HT29: sh-DLEU2 + sh-NC vs. sh-DLEU2 + sh-RARB: *p* = 0.0006). The apoptosis of CRC cells was reduced after RARB downregulation (Figure 6e) (SW480: sh-DLEU2 + sh-NC vs. sh-DLEU2 + sh-RARB: *p* = 0.0001; HT29: sh-DLEU2 + sh-NC vs. sh-DLEU2 + sh-RARB: *p* = 0.0003). Moreover, the phosphorylation of Raf, p38, and ERK in cells was elevated after RARB silencing (figure 6f) (see *p* values in Table 4). Moreover, the cells transfected with oe-DLEU2 were treated with Dehydrocorydaline, after which the phosphorylation of p38 in cells was significantly elevated (Figure 6g) (SW480: sh-DLEU2 + DMSO vs. sh-DLEU2 + Dehydrocorydaline: *p* = 0.0006; HT29: sh-DLEU2 + DMSO vs. sh-DLEU2 + Dehydrocorydaline: *p* = 0.0052). In this setting, the proliferation of cells was significantly restored (Figure 6h) (sh-DLEU2 + DMSO vs. sh-DEU2 + Dehydrocorydaline: SW480: 0 h: *p* = 0.9990, 24 h: *p* = 0.6695, 48 h: *p* < 0.0001, 72 h *p* < 0.0001; HT29: 0 h, *p* = 0.9997, 24 h: *p* = 0.0603, 48 h: *p* < 0.0001, 72 h, *p* < 0.0001). Moreover, the migration (Figure 6i) (sh-DLEU2 + DMSO vs. sh-DEU2 + Dehydrocorydaline: SW480: *p* < 0.0001; HT29: *p* < 0.0001) and invasiveness (Figure 6j) (sh-DLEU2 + DMSO vs. sh-DEU2 + Dehydrocorydaline: SW480: *p* = 0.001; HT29: *p* = 0.0017). The Dehydrocorydaline treatment also reduced the apoptosis rate of cells (Figure 6k) (sh-DLEU2 + DMSO vs. sh-DEU2 + Dehydrocorydaline: SW480: *p* = 0.0005; HT29: *p* = 0.0004).

RETRACTED

**Figure 6.** RARB silencing blocks the inhibiting role of sh-DLEU2 in CRC cells. (a) RARB expression in SW480 and HT29 cells after sh-RARB transfection detected by RT-qPCR (DLEU2: SW480: sh-DLEU2 + sh-NC vs. sh-DLEU2 + sh-RARB: *p* = 0.9657; HT29: sh-DLEU2 + sh-NC vs. sh-DLEU2 + sh-RARB: *p* = 0.8714; RARB: SW480: sh-DLEU2 + sh-NC vs. sh-DLEU2 + sh-RARB: *p* = 0.0006; HT29: sh-DLEU2 + sh-NC vs. sh-DLEU2 + sh-RARB: *p* = 0.0001); (b) viability of SW480 and HT29 cells examined by the CCK-8 method (two-way ANOVA) (SW480: 0 h: *p* = 0.9931; 24 h: *p* = 0.4837; 48 h: *p* = 0.0069; 72 h: *p* = 0.0001; HT29: 0 h: *p* = 0.9947; 24 h: *p* = 0.2835; 48 h: *p* = 0.0013; 72 h: *p* < 0.0001); (c-d) migration and invasiveness of SW480 and HT29 cells measured by Transwell assays, respectively (two-way ANOVA) (C: SW480: sh-DLEU2 + sh-NC vs. sh-DLEU2 + sh-RARB: *p* = 0.0005; HT29: sh-DLEU2 + sh-NC vs. sh-DLEU2 + sh-RARB *p* = 0.0002; D: SW480: sh-DLEU2 + sh-NC vs. sh-DLEU2 + sh-RARB: *p* = 0.001; HT29: sh-DLEU2 + sh-NC vs. sh-DLEU2 + sh-RARB: *p* = 0.0006); (e) apoptosis of SW480 and HT29 cells detected by flow cytometry (two-way ANOVA) (SW480: sh-DLEU2 + sh-NC vs. sh-DLEU2 + sh-RARB: *p* = 0.0001; HT29: sh-DLEU2 + sh-NC vs. sh-DLEU2 + sh-RARB: *p* = 0.0003); (f) phosphorylation and protein levels of Raf, p38, and ERK in CRC cells determined by immunoblot analysis (two-way ANOVA) (see *p* values in Table 4); (g) p38 phosphorylation in CRC cells after Dehydrocorydaline treatment examined by immunoblot analysis (sh-DLEU2 + DMSO vs. sh-DLEU2 + Dehydrocorydaline: SW480: *p* = 0.0006; HT29: *p* = 0.0052); (h) proliferation of cells examined by the CCK-8 assay (sh-DLEU2 + DMSO vs. sh-DEU2 + Dehydrocorydaline: SW480: 0 h: *p* = 0.9990, 24 h: *p* = 0.6695, 48 h: *p* < 0.0001, 72 h: *p* < 0.0001; HT29: 0 h, *p* = 0.9997, 24 h: *p* = 0.0603, 48 h: *p* < 0.0001, 72 h, *p* < 0.0001); (i-j) migration (i, sh-DLEU2 + DMSO vs. sh-DEU2 + Dehydrocorydaline: SW480: *p* < 0.0001; HT29: *p* < 0.0001) and invasiveness (j, sh-DLEU2 + DMSO vs. sh-DEU2 + Dehydrocorydaline: SW480: *p* = 0.001; HT29: *p* = 0.0017) of cells analyzed by Transwell assays; (k) apoptosis of cells examined by flow cytometry (sh-DLEU2 + DMSO vs. sh-DEU2 + Dehydrocorydaline: SW480: *p* = 0.0005; HT29: *p* = 0.0004). Repetition = 3.

RETRACTED

**Table 4.** *P* values of the phosphorylation extent of the Raf, p38, and ERK between the sh-DLEU2 + sh-NC and sh-DLEU2 + sh-RARB groups in SW480 and HT29 cells

Cell lines	Protein	Data comparisons	*P* values
SW480	p-Raf	sh-DLEU2 + sh-NC vs. sh-DLEU2 + sh-RARB	*p* = 0.0185
	Raf	sh-DLEU2 + sh-NC vs. sh-DLEU2 + sh-RARB	*p* = 0.997
	p-p38	sh-DLEU2 + sh-NC vs. sh-DLEU2 + sh-RARB	*p* = 0.02
	p38	sh-DLEU2 + sh-NC vs. sh-DLEU2 + sh-RARB	*p* > 0.9999
	p-ERK	sh-DLEU2 + sh-NC vs. sh-DLEU2 + sh-RARB	*p* = 0.0031
	ERK	sh-DLEU2 + sh-NC vs. sh-DLEU2 + sh-RARB	*p* = 0.997
HT29	p-Raf	sh-DLEU2 + sh-NC vs. sh-DLEU2 + sh-RARB	*p* = 0.0164
	Raf	sh-DLEU2 + sh-NC vs. sh-DLEU2 + sh-RARB	*p* = 0.984
	p-p38	sh-DLEU2 + sh-NC vs. sh-DLEU2 + sh-RARB	*p* = 0.0222
	p38	sh-DLEU2 + sh-NC vs. sh-DLEU2 + sh-RARB	*p* > 0.9999
	p-ERK	sh-DLEU2 + sh-NC vs. sh-DLEU2 + sh-RARB	*p* = 0.0127
	ERK	sh-DLEU2 + sh-NC vs. sh-DLEU2 + sh-RARB	*p* > 0.9999

## Discussion

The epigenetic regulation exerts essential functions in the tumorigenesis of CRC, a tumor with a strong epigenetic component that drives malignant transformation of cancer cells earlier than other genetic changes [33]. In this paper, we confirmed that DLEU2 induces promoter methylation and loss of expression of the tumor inhibitor RARB and enhanced viability and mobility of CRC cells through the activation of the MAPK pathway.

Advance in bioinformatic technologies has allowed the development of new genomic landscape including lncRNAs and revealed their versatile functions and important involvements in the progression of cancers through interacting with other cellular molecules [34]. In the present study, we identified four significantly differentially expressed lncRNAs in CRC including CRNDE, LINC00460, PVT1, and DLEU2 by analyzing three GEO datasets GSE146587, GSE156720, and GSE184093. Both CRNDE [35], LINC00460 [36], PVT1 [37] have been reported to play oncogenic roles in CRC with the interacted molecules clearly defined. Although DLEU2 has also been found to induce the proliferation and invasiveness of CRC [13], the molecular mechanisms remain largely unknown. Activation of DLEU2 has been correlated with tumorigenesis of several malignancies, such as gastric cancer [38] and cervical cancer [39], by regulating the NOTCH signaling pathway. In this work, we identified the high-expression pattern of DLEU2 in CRC cell lines compared to normal FHC cells, and the DLEU2 knockdown in cancer cells suppressed proliferation, invasiveness, and resistance to death of cells. These findings validate the tumor-promoting roles of DLEU2 in CRC.

RETRACTED

As it can be seen in several examples above that a major mechanism by which lncRNAs exert their bioinformatic functions is that when locate in cytoplasm, they may work as competing endogenous RNAs (ceRNAs) and diminish the binding effect of miRNA on its downstream mRNAs [40]. For DLEU2, it has been suggested to trigger tumorigenesis via such ceRNA networks [41,42]. However, our FISH and nuclear-cytoplasmic RNA separation assays confirmed a nuclear localization of DLEU2 in CRC cells. In this case, lncRNAs may function as epigenetic modulators that modulate chromatin states and impacting gene expression [8,43]. Our microarray analysis suggested that RARB was significantly upregulated in cells with DLEU2 knockdown and the subsequent qMSP assay identified increased DNA methylation at the RARB promoter. As aforementioned, lncRNAs may recruit, sequester, or regulate expression of DNMTs to regulate DNA methylation in downstream genes [15]. A recent publication by Zhang *et al*., for instance, reported that lncRNA LALC recruits DNMTs to LZTS1 promoter to suppress its expression, which facilitated liver metastasis of CRC [44]. The lincRNA DACOR1 was found to reprogram the genome-wide DNA methylation pattern in colon cancer [45,46]. In this work, our RIP and ChIP results identified that DLEU2 suppresses RARB expression by inducing DNMT1-mediated DNA methylation. RARB is a tumor inhibitor protein involved in cell proliferation and differentiation, cell cycle progression, and apoptosis [47]. RARB downregulation is associated with retinoid resistance and tumorigenesis, whereas induction of RARB can suppress cancer progression [48]. Hypermethylation of RARB has been indicated as a possible biomarker for lung cancer [20], breast cancer [19], prostate cancer [49]. Likewise, hypermethylation of RARB has been observed in CRC [50]. We observed that further silencing of RARB rescued the proliferation and invasiveness of CRC cells suppressed by sh-DLEU2. The RARB targets were largely enriched in the MAPK signaling according to our KEGG pathway enrichment analysis. The MAPK pathway is one of the best-recognized pathways in tumorigenesis whose hyperactivation is associated with over 40% human cancer cases and drives tumor formation by activating proliferative genes and overcoming metabolic stress [51]. MAPKs react to a multitude of input signals, and they are traditionally allocated in mitogen responsive MAPKs (ERK) and stress responsive MAPKs (JNK and p38) [52]. Molecules of this signaling cascade are master regulators of cell apoptosis [53]. Activation of the MAPK signaling pathway has also been implicated in the tumorigenesis of CRC [54]. Importantly, we observed that the phosphorylation of Raf, p38, and ERK in CRC cells was reduced upon DLEU2 silencing but restored after further RARB inhibition. In agreement with this, RARB was found to suppresses MAPK kinase kinase 2 to inactivate the MAPK signaling, and the RARB downregulation by miRNA-106a led to MAPK activation and increased the apoptosis of thyroid cancer cells [55]. Moreover, we found that treatment with the p38-specific agonist Dehydrocorydaline restored the proliferation, whereas suppressed the apoptosis of cancer cells induced by DLEU2 knockdown, which confirmed that the DLEU2/RARB axis regulates CRC tumorigenesis by manipulating the MAPK signaling pathway.

RETRACTED

## Conclusion

In conclusion, this study demonstrates that DLEU2 augments CRC progression by inducing DNMT1-mediated RARB promoter methylation and activating the MAPK signaling pathway. This study suggests that DLEU2 may serve as a diagnostic marker and a potential target for CRC treatment. However, amongst the many downstream molecules of the MAPK pathway, we did not define the exact factors responsible for the DLEU2/RARB cascade-mediated malignant phenotype of CRC cells. We would like to figure this out in our future researches.

## Supplementary Material

Supplemental Material

## Data Availability

All the data generated or analyzed during this study are included in this published article.
